# Construction of a Prognostic Nomogram Model for Patients with Mucinous Breast Cancer

**DOI:** 10.1155/2022/1230812

**Published:** 2022-03-23

**Authors:** Xulong Zhu, Ying Li, Fende Liu, Feifei Zhang, Jianhui Li, Chong Cheng, Yanwei Shen, Nan Jiang, Jia Du, Yajing Zhou, Binliang Huo

**Affiliations:** ^1^Department of Surgical Oncology, Shaanxi Provincial People's Hospital, Xian 710068, China; ^2^School of Life Science and Technology, Xi'an Jiaotong University, Xi'an 710049, China; ^3^Graduate School, Xi'an Medical University, Xi'an 710068, China

## Abstract

**Objective:**

The objective of the study is to develop a nomogram for estimating three- and five-year survival rates in mucinous breast cancer patients.

**Methods:**

Between 2010 and 2016, the National Cancer Institute's Surveillance, Epidemiology, and End Results (SEER) were searched as a data source for patients associated with mucinous breast cancer (MBC). A total of 3964 patients were recruited after screening. The multivariate Cox model and the univariate Kaplan-Meier (KM) approach were employed to evaluate the independent prognostic markers, followed by developing a nomogram for estimating three- and five-year survival rates in MBC patients. Consequently, the consistency index (C-index) was employed to assess the predictive accuracy of the generated nomogram.

**Results:**

Age, race, T stage, M stage, surgery, and radiotherapy were all independent predictive biomarkers for the MBC patients (*P* < 0.05). The nomogram was finally developed based on the underlined factors. Furthermore, the C-index of 0.803 and reliable calibration curves were obtained in the nomogram's assessment.

**Conclusions:**

In patients with mucinous breast cancer, the proposed nomogram provides a viable tool for accurate prognostic prediction. In clinical practice, it could serve as a personalized diagnosis tool, estimate prognosis, and help in suggesting treatment plans for patients with MBC.

## 1. Introduction

Mucinous breast cancer (MBC) is a rare and unusual type of breast cancer that manifests itself primarily by a huge percentage of extracellular mucins [1, 2]. It accounts for around 1%–6% of all primary breast cancers. MBC is more frequent in postmenopausal women and has a better survival [3]. MBC was shown to have elevated hormone receptor expression and decreased human epidermal growth factor receptor 2 expressions in prior research [4–6]. Because of the low incidence of MBC, it has different clinical, histopathological, and biological characteristics from common breast cancers in general [7], and there is a lack of reports of large sample studies on MBC, which predisposes to undertreatment or overtreatment. The prognosis of MBC is influenced by many factors at the same time. It is difficult to predict the actual situation of patients by one or several prognostic factors alone. The lack of a particular prognosis evaluation system for MBC has resulted in a uniform treatment for MBC, without any consideration of individual patient needs.

Nomograms have been developed as the new standard for predicting the occurrence and prognosis of certain cancers, and most cancer types have established prognostic nomograms [8, 9]. Such nomograms are considered a reliable tool that can help clinicians make accurate individualized predictions [10]. However, no satisfactory nomogram has yet been developed to predict survival in MBC. To solve the problem, this study attempts to establish a new nomogram-based prediction model for MBC that incorporates more than one clinical parameter in an attempt to individualize the estimation of prognosis for patients. It involves retrospective analysis of the data of MBC from 2010 to 2016 in the SEER database, screening independent prognostic factors, and, subsequently, constructing a nomogram prognostic model to provide a reference for clinicians to assess patient prognosis and develop individualized treatment plans.

## 2. Material and Methods

### 2.1. Source of Data

The data for the current study were attained from the SEER database of the US National Cancer Institute (NCI), and the data were obtained by SEER Stat 8.3.8 software.

### 2.2. Patient Inclusion and Information Extraction

#### 2.2.1. Patient Inclusion and Exclusion Criteria

The data of MBC patients in the SEER database from 2010 to 2016 were collected. Inclusion criteria were as follows: (1) ICD-O-3 Hist/behave, malignant = “8480/3: mucinous adenocarcinoma”; (2) patients newly diagnosed with MBC; (3) patients with breast cancer as the only primary tumor; (4) patients with complete general clinicopathological information; (5) patients with complete follow-up (follow-up up to December 31, 2016). The exclusion criteria were given as follows: (1) male MBC patients; (2) confirmed patients of postmortem examination and death report; (3) patients with missing information and survival time less than 1 month (Figure 1).

#### 2.2.2. Information Extraction

Extract the patient's age, race, marital status, tumor location (left breast, right breast), histological grade, TNM stage (7th edition AJCC-TNM staging system), ER status, PR status, HER-2 status, surgery, radiotherapy, chemotherapy, survival data, and other information.

### 2.3. Statistical Methods

Patients were randomly split into modeling and validation groups using *R* software. First, univariate analysis was conducted to evaluate the factors affecting the survival prognosis of patients in the modeling group, and variables that showed statistical significance on univariate analysis were also involved in the multivariate Cox proportional hazards regression (CPHR) model to determine the final independent prognostic factors, the effect of independent prognostic factors on the survival rate of MBC patients was shown by the KM method, and then, the nomogram was constructed using *R* software, and the consistency index was calculated, and the correction curve was drawn. The Bootstrap method was used to conduct internal and external validation for the modeling group and the validation group, respectively. In the calibration curve, the closer the curve is to the ideal 45° reference line, the closer the predicted value is to the actual observed value. *R* software (version 4.0.2) (http://www.r-project.org/) was employed to conduct the statistical evaluations.

## 3. Results

### 3.1. Clinicopathological Features of Included Patients

From 2010 to 2016, the SEER database yielded 3,964 eligible female MBC patients (2,776 in the modeling group and 1,188 in the validation group). It summarizes the sociodemographic and clinicopathological features of the two groups in Table 1. The 3,964 patients were followed up for a period of 1 to 83 months, with a mean follow-up of 39 months. Approximately three-quarters of patients were white (*n* = 2,992, 75.4%), more than one-half were Grade I (*n* = 2,354, 59.3%), and more than 90% were N0, M0, ER (+), PR (+), HER-2 (−). Other clinicopathological features are shown in Table 1.

### 3.2. Analysis of Influencing Factors of Survival Prognosis

#### 3.2.1. Univariate Analysis Results

Univariate analysis of the survival of 2,776 MBC patients in the modeling group revealed that the 3- and 5-year survival rates of patients were linked to their age, ethnicity, marital status, T stage, N stage, M stage, surgery, radiotherapy, and chemotherapy (*P* < 0.05) but not to histological grade, lesion location, PR status, ER status, or HER-2 status (*P* > 0.05), as indicated in Table 2.

#### 3.2.2. Results of Multivariate CPHR Analysis

Table 2 shows the results of multivariate CPHR analysis, which were based on the findings of univariate analysis. In this study, age, ethnicity, T stage, M stage, surgery, and radiotherapy were all found to be independent risk factors for MBC patients' prognosis (*P* < 0.05). The KM curve was used to demonstrate the impact of independent prognostic factors on MBC patient survival rates, as indicated in Figures 2(a)–2(f). In each of the graphical representations, the horizontal axis (*x*-axis) represents time in months, and the vertical axis (*y*-axis) shows the probability of survival or the proportion of people surviving. A vertical drop in the curves indicates an event.

### 3.3. The Development of a Nomogram to Assess MBC Patients' 3- and 5-Year Overall Survival (OS) Rates

Age, ethnicity, T stage, M stage, radiation, and surgery were among the statistically significant prognostic factors in the multivariate CPHR model. A nomogram was constructed using *R* software. The predictive nomogram for the 3- and 5-year OS rates of MBC patients is shown in Figure 3. The nomogram is used by totaling the points identified on the top scale for each independent covariate. The score of each item of an individual can be obtained by projecting each clinicopathologic feature upwards to the score, and the total score is obtained by adding the scores of each item. There is a total points line at the bottom of the nomogram. The total points projected to the bottom scale indicate the % probability of 3-, 5-year ***overall survival (OS).***

The higher the total score, the worse the survival prognosis. The nomogram in Figure 3 shows that age at diagnosis is the greatest contributor to the prognosis, followed, respectively, by M stage, TNM stage, ethnicity, surgery status, and radiotherapy status. The nomogram shows that the use of radiotherapy is beneficial for patients with MBC.

### 3.4. Verification of Nomograms

We established a nomogram model integrating independent predictors of OS (e.g., age, tumor site, tumor size, tumor extension, and radiotherapy) to provide a visual statistical predictive tool for the survival of patients with MGCTB. We established a nomogram model integrating independent predictors of OS (e.g., age, tumor site, tumor size, tumor extension, and radiotherapy) to provide a visual statistical predictive tool for the survival of patients with MGCTB. We established a nomogram model integrating independent predictors of OS (e.g., age, tumor site, tumor size, tumor extension, and radiotherapy) to provide a visual statistical predictive tool for the survival of patients with MGCTB. We established a monogram model integrating independent predictors of OS (age, ethnicity, T stage, M stage, radiotherapy, and surgery) to provide a visual statistical predictive tool for the survival of patients with MBC. A calibration curve of the nomograph was drawn to evaluate the consistency between the observed and estimated survivals. The C-index calculated by *R* software was 0.803 (95% CI: 0.772–0.834) for the modeling group and 0.817 (95% CI: 0.768–0.866) for the validation group, suggesting that both had good predictive values and good discriminative ability. The bootstrap method was used for internal verification and external verification of nomogram. The self-sampling number *B* = 1,000.  Figure 4 shows the calibration plots of the nomogram for predicting the probability of OS at 3 and 5 years. The calibration curves of 3- and 5-year survival rates in the modeling group and validation group were close to the ideal 45° reference line (Figure 4), suggesting that there was good consistency between the predicted value and the actual 3 and 5 years OS. Thus, the monogram has been internally and externally verified for both the modeling and validation group, respectively, showing good accuracy and clinical applicability. It can effectively predict OS in MBC patients, which may help clinicians personalize prognostic assessments and clinical decisions.

## 4. Discussions

MBC is a kind of breast cancer that is quite uncommon. It affects 1%–6% of all initial breast tumors. [1, 11] Relative to other kinds of breast cancer, MBC has a few distinct clinical characteristics. MBC is more common in postmenopausal and elderly women and has a satisfactory rate of survival. The positive rates of estrogen and progesterone receptors in MBC are substantial and demonstrate greater differentiation and a decreased rate of lymph node metastasis [6, 12, 13]. The underlined data showed consistency with the findings of this study. Because of its rarity in the clinic, most studies on MBC have small sample sizes, relatively short follow-up times, and insufficient evidence on the clinical influencing factors and survival of MBC patients. Currently, data from invasive ductal carcinoma are used to generate guideline recommendations for both local and systemic adjuvant treatment of MBC, and the accuracy of survival prognostic information is influenced by physician experience, so a more accurate survival prediction model is lacking. In this study, an objective nomogram was constructed based on the SEER database to make a more accurate estimate of the 3- and 5-year survival rates of patients suffering from MBC, which improved the rationality of both doctors and patients for disease management and was important for clinical decision-making.

In this study, we analyzed multiple possible prognostic factors in MBC patients, and the results showed that age, ethnicity, T stage, M stage, surgery, and radiotherapy were all independent factors for patient survival prognosis. In our study, 68.1% of patients were over 60 years of age, and the prognosis was best for people aged 40–59 years, and previous studies have shown that MBC is common in older patients, and its incidence generally peaks after menopause [6, 14]. Patients with MBC had high ER or PR positivity (98.8% and 92.0% of ER and PR positivity, accordingly), low histological score (59.3% Grade I), and less lymph node metastasis (90.1% without lymph node metastasis). The findings of this study were consistent with the findings of previous research [2, 5, 15–17], which demonstrated that MBC patients had a substantial chance of surviving.

The predictive importance of tumor size in MBC patients is a point of contention. Patients with tumors greater than 2 cm were previously advised to take adjuvant chemotherapy, according to NCCN recommendations. However, the recommendations have been modified so that only lymph node involvement is considered chemotherapeutic, regardless of the T stage. While tumor size has been linked to the diagnosis of less aggressive tumors, its predictive value has been questioned due to the inclusion of extensive extracellular mucins in tumor size measurement [18]. As a result, tumor size measurements may not accurately reflect actual tumor size, making tumor size prediction problematic [19]. Furthermore, lymph node involvement was found to be unrelated to tumor size in one investigation [20]. T3 and T4 tumors had a worse prognosis than T1 and T2 tumors in our study, according to the nomogram. As a result, a tumor with a diameter of more than 5 cm may be associated with a bad prognosis.

At present, the treatment modalities for MBC patients are mainly surgery, chemotherapy, radiotherapy, and endocrine therapy. The choice of surgical approach also has a considerable influence on the subsequent treatment options of patients and the survival prognosis of patients. In this study, 3,817 patients (96.2%) received surgical treatment, and the nomogram showed that the prognosis of patients who received surgical treatment was better than that of patients who did not receive surgery. It has been shown that patients treated with breast-conserving surgery in stage T1-2 MBC have a better prognosis than those who undergo mastectomy, particularly in patients aged 50–79 years; [21] however, this study did not compare the specific modalities of surgery, and in the subsequent study, we will consider this aspect of the influencing factors. As a considerable adjuvant therapy, radiotherapy is commonly used in patients with high-risk factors post breast-conserving therapy or mastectomy for breast cancer [22]. However, there is a lack of clarity regarding the clinical value of radiotherapy in MBC. In the current study, a total of 2,043 (51.5%) patients received radiotherapy and 1,921 (48.4%) did not. The nomogram shows that the use of radiotherapy is beneficial for patients with MBC. It has been reported in the literature that [23, 24] the reason for the low efficacy of chemotherapy is that mucus accounts for most of the total volume in MBC cells, forming a large pool of mucin, resulting in inconsistency between clinical or imaging assessment of chemotherapy efficacy and mucinous carcinoma pathology. Despite the effective elimination of malignant cells by chemotherapy, the mucin pool remains [25].

However, this study has several limitations. First, important details such as treatment information (e.g., radiation dose, chemotherapy dose, targeted therapy, endocrine therapy, or immunotherapy) are missing in the SEER database because most patients with MBC are hormone receptor-positive. Patients who complete local therapy are likely to receive standard endocrine therapy, and the SEER database cannot provide data on endocrine therapy and is difficult to guide physicians in the treatment of patients of the same category. Second, the lack of information in the SEER database may affect the data of the CPHR model (such as Ki-67, tumor markers, and other related factors), and these important variables should be considered in future studies. Finally, the database does not perform specific pathological classification of MBC, such as pure mucinous breast carcinoma (PMBC) as well as mixed mucinous breast carcinoma (MMBC) [26], because MBC of different pathological types may have different prognoses. The nomograms in this study were internally and externally validated for the population of the SEER database. It is validated in the same population, and the validation of model performance can be biased. Hence, other multicenter data are needed for external validation to further test the predictive effect of nomograms.

## 5. Conclusion

Routine clinical data obtained from the SEER database were used to develop a useful clinical nomogram that could help clinicians treat MBC in their daily practice. The nomogram incorporates various clinicopathological indicators and can render great help in clinical decision-making thereby enabling individualized therapy and management of MCB patients.

The future directions of this work will potentially involve a larger sample size, including more related factors to further screen the independent influencing factors of the prognosis of MBC patients. In addition, we plan to carry out a multicenter prospective randomized controlled study to verify its predictive effect, improve the nomogram prognostic model, and provide a reference for the evaluation of the prognosis of MBC patients as well as the selection of personalized treatment plan.

## Figures and Tables

**Figure 1:** Flow chart of patient screening in SEER database.

**Figure 2:** Kaplan-Meier curve of the effect of each independent risk factor on the prognosis of MBC. (a) Age; (b) ethnicity; (c) T stage; (d) M stage; (e) with or without surgery; (f) with or without radiotherapy.

**Figure 3:** Prognostic nomogram models for 3- and 5-year OS rates of MBC patients. The nomogram is used by totaling the points identified on the top scale for each independent covariate. The total points projected to the bottom scale indicate the % probability of 3- and 5-year OS.

**Figure 4:** Calibration curve of the nomogram for predicting the probability of OS at 3 and 5 years. (a, b) modeling group; (c, d) validation group.

**Table 1:** Clinicopathological features of patients in modeling and validation group (case (%)).

Clinicopathological characteristics	Modeling group (*n* = 2776)		Validation group (*n* = 1188)	
Age				
18–39	116	4.1	44	3.7
40–59	772	27.8	326	27.4
60–79	1448	52.1	605	50.9
≥80	440	15.8	213	17.9
Ethnicity				
White	2087	75.1	905	76.1
Black	343	12.3	144	12.1
Others	346	12.4	139	11.7
Marital status				
Married	1418	51.0	608	51.1
Unmarried	1358	48.9	580	48.8
Lesion location				
Left	1435	51.6	616	51.8
Right	1341	48.4	572	48.1
Histological grading				
I	1644	59.2	710	59.7
II	1030	37.1	428	36.0
III	100	3, 6	49	4.1
IV	2	0.1	1	0.1
T Stage				
T1	1776	63.9	795	66.9
T2	798	28.7	322	27.1
T3	153	5.5	56	4.7
T4	49	1.7	15	1.2
N Stage				
N0	2506	90.2	1068	89.8
N1	216	7.7	101	8.5
N2	32	1.1	16	1.3
N3	22	0.7	3	0.2
M Stage				
M0	2741	98.7	1174	98.8
M1	35	1.2	14	1.1
ER expression				
Negative	36	1.2	10	0.8
Positive	2740	98.7	1178	99.1
PR expression				
Negative	213	7.6	104	8.7
Positive	2563	92.3	1084	91.2
HER-2 expression				
Negative	2614	94.1	1131	95.2
Positive	162	5.8	57	4.7
Surgery				
Yes	2667	96.0	1150	96.8
None	109	3.9	38	3.1
Radiotherapy				
Yes	1419	51.1	624	52.5
None	1357	48.8	564	47.4
Chemotherapy				
Yes	381	13.7	157	13.2
None	2395	86.2	1031	86.7

**Table 2:** Results of univariate and multivariate analysis affecting the survival prognosis of 2776 patients in the modeling group.

Clinical pathology characteristics	Univariate analysis			Multivariate analysis		
	Hr value	95% confidence interval	*P* Value	HR value	95% confidence interval	*P* Value
Age						
18–39		1			1	
40–59	0.92	0.32–2.66	0.892	0.75	0.26 to 2.19	0.604
60–79	1.73	0.63–4.71	0.285	1.61	0.57–4.52	0.368
≥80	7.67	2.83–20.81	<0.001	5.34	1.89–15.08	0.002
Ethnicity						
White		1			1	
Black	1.07	0.73 to 1.57	0.725	1.17	0.79–1.74	0.434
Others	0.39	0.22–0.70	0.001	0.48	0.26 to 0.87	0.015
Marital status						
Married		1			1	
Unmarried	2.10	1.60–2.77	<0.001	1.22	0.91 to 1.64	0.184
Lesion location						
Left		1			1	
Right	1.14	0.88–1.48	0.311	1.88	0.91 to 1.55	0.205
Histological grading						
I		1			1	
II	1.09	0.83–1.44	0.522	1.00	0.76–1.33	0.978
III	1.62	0.90–2.93	0.110	1.98	0.63–2.28	0.584
IV	4.79	0.67–34.29	0.119	2.29	0.30–17.59	0.427
T Stage						
T1		1			1	
T2	1.93	1.45–2.57	<0.001	1.69	1.25–2.30	<0.001
T3	2.53	1.58–4.04	<0.001	1.77	1.05–2.97	0.031
T4	9.72	5.88–16.07	<0.001	3.54	1.86–6.73	<0.001
N Stage						
N0		1			1	
N1	1.60	1.06–2.41	0.025	1.37	0.88–2.15	0.168
N2	2.13	0.87–5.18	0.095	2.16	0.84–5.56	0.111
N3	3.71	1.52–9.02	0.039	0.35	0.12–1.07	0.066
M Stage						
M0		1			1	
M1	12.10	7.69–19.05	<0.001	7.22	3.98–13.12	<0.001
ER expression						
Negative		1			1	
Positive	0.72	0.27–1.93	0.514	0.70	0.23–2.11	0.529
PR expression						
Negative		1			1	
Positive	0.68	0.45–1.02	0.065	0.77	0.49 to 1.21	0.257
HER-2 expression						
Negative		1			1	
Positive	0.56	0.28–1.23	0.105	1.02	0.48–2.19	0.956
Surgery						
Yes		1			1	
None	6.69	4.59–9.76	<0.001	1.96	1.22–3.13	0.005
Radiotherapy						
Yes		1			1	
None	2.86	2.15–3.82	<0.001	1.86	1.37–2.51	<0.001
Chemotherapy						
Yes		1			1	
None	1.79	1.12–2.86	0.015	1.41	0.78–2.55	0.250

## Data Availability

Data will be provided on request.

## References

[1] Naqos N., Naim A., Jouhadi H. (2016). Mucinous carcinoma of the breast: clinical, biological and evolutive profile. *Cancer Radiotherapie*.

[2] Skotnicki P., Sas-Korczynska B., Strzepek L. (2016). Pure and mixed mucinous carcinoma of the breast: a comparison of clinical outcomes and treatment results. *Breast Journal*.

[3] Diab S. G., Clark G. M., Osborne C. K., Libby A., Allred D. C., Elledge R. M. (1999). Tumor characteristics and clinical outcome of tubular and mucinous breast carcinomas. *Journal of Clinical Oncology*.

[4] SAUDADE, André F. E. R. N. A. N. D. O. (1995). Mucinous carcinoma of the breast: a pathologic study of 82 cases. *Journal of Surgical Oncology*.

[5] Louwman M. W. J., Vriezen M., Beek M. W. P. M. V. (2010). Uncommon breast tumors in perspective: incidence, treatment and survival in The Netherlands. *International Journal of Cancer Journal International Du Cancer*.

[6] Di Saverio S., Gutierrez J., Avisar E. (2008). A retrospective review with long term follow up of 11,400 cases of pure mucinous breast carcinoma. *Breast Cancer Research and Treatment*.

[7] Ha K. Y., Deleon P., Deleon W. (2013). Invasive mucinous carcinoma of the breast. *Baylor University Medical Center Proceedings*.

[8] Huang Y.-q., Liang C.-h., He L. (2016). Development and validation of a radiomics nomogram for preoperative prediction of lymph node metastasis in colorectal cancer. *Journal of Clinical Oncology*.

[9] Liang W., Zhang L., Jiang G. (2015). Development and validation of a nomogram for predicting survival in patients with resected non-small-cell lung cancer. *Journal of Clinical Oncology*.

[10] Corso G., Maisonneuve P., Massari G. (2020). Validation of a novel nomogram for prediction of local relapse after surgery for invasive breast carcinoma. *Annals of Surgical Oncology*.

[11] Ohashi R., Sakatani T., Matsubara M. (2016). Mucinous carcinoma of the breast: a comparative study on cytohistological findings associated with neuroendocrine differentiation. *Cytopathology*.

[12] Bae S. Y., Choi M. Y., Cho D. H. (2011). Mucinous carcinoma of the breast in comparison with invasive ductal carcinoma: clinicopathologic characteristics and prognosis. *Journal of Breast Cancer*.

[13] Tseng H.-S., Lin C., Chan S.-E. (2013). Pure mucinous carcinoma of the breast: clinicopathologic characteristics and long-term outcome among Taiwanese women. *World Journal of Surgical Oncology*.

[14] Li C. I. (2010). Risk of mortality by histologic type of breast cancer in the United States. *Hormones and Cancer*.

[15] Hanagiri T., Ono K., Baba T. (2010). Clinicopathologic characteristics of mucinous carcinoma of the breast. *International Surgery*.

[16] Avisar E., Khan M. A., Axelrod D., Oza K. (1998). Pure mucinous carcinoma of the breast: a clinicopathologic correlation study. *Annals of Surgical Oncology*.

[17] Fentiman I., Millis R., Smith P., Ellul J., Lampejo O. (1997). Mucoid breast carcinomas: histology and prognosis. *British Journal of Cancer*.

[18] Kim D., Jung W.-H., Koo J. S. (2012). Expression of MUC1, MUC2, MUC5AC and MUC5B in mucinous lesions of the breast. *Pathobiology*.

[19] Ranade A., Batra R., Sandhu G., Chitale R. A., Balderacchi J. (2010). Clinicopathological evaluation of 100 cases of mucinous carcinoma of breast with emphasis on axillary staging and special reference to a micropapillary pattern. *Journal of Clinical Pathology*.

[20] Paramo J. C., Wilson C., Velarde D., Giraldo J., Poppiti R. J., Mesko T. W. (2002). Pure mucinous carcinoma of the breast: is axillary staging necessary?. *Annals of Surgical Oncology*.

[21] Yu P., Liu P., Zou Y. (2020). Breastヽonserving therapy shows better prognosis in mucinous breast carcinoma compared with mastectomy: a SEER population‐based study. *Cancer Medicine*.

[22] Bernard F. (2002). Twenty-year follow-up of a randomized trial comparing total mastectomy, lumpectomy, and lumpectomy plus irradiation for the treatment of invasive breast cancer. *New England Journal of Medicine*.

[23] Von Minckwitz G., Costa S. D., Eiermann W. (1999). Maximized reduction of primary breast tumor size using preoperative chemotherapy with doxorubicin and docetaxel. *Journal of Clinical Oncology*.

[24] Lannigan A. K., Going J. J., Weiler-Mithoff E., Cooke T. G. (2002). Mucinous breast carcinoma. *The Breast*.

[25] Didonato, Rosemarie S. H. A. P. I. R. O. (2018). *Invasive Mucinous Carcinoma of the Breast and Response Patterns after Neoadjuvant Chemotherapy (NAC)*.

[26] Kashiwagi S., Onoda N., Asano Y. (2013). Clinical significance of the sub-classification of 71 cases mucinous breast carcinoma. *SpringerPlus*.

